This article has been retracted.

# The Effect of Mental Health Intervention before English Test on College Students' English Test Scores

**DOI:** 10.1155/2022/4998180

**Published:** 2022-09-10

**Authors:** Yan Sun

**Affiliations:** School of Foreign Languages, Zhengzhou University of Aeronautics, Zhengzhou Henan 450046, China

## Abstract

It is necessary to pay attention to and study the physical and mental health development of college students. On the basis of statistical analysis of the questionnaire, this paper studies the impact of pretest mental health intervention on college students' English test scores, summarizes the problems and characteristics of college students' mental health, and explores the reasons for psychological problems. Based on the research results and related survey data of the mental health status of college students by scholars, this paper believes that these reasons mainly include students' personal reasons, school and social environment pressure, and insufficient family support factors. The data analysis shows that in the relationship between English education and mental health in colleges and universities, the amount of mental health intervention of students' extracurricular exercise has a stable and low negative correlation with the scores of each factor of SCL-90 (Symptom Checklist 90) and is negatively correlated with the scores of each subscale. The experimental results show that there are extremely significant differences in academic performance (*F* = 5.084, *P* < 0.01), and there is a certain linear relationship between students' mental health level and students' English exercise feeling. The lower the fatigue score, the higher the mental health level of the students, which effectively promotes the mental health development of college students.

## 1. Introduction

As the trend of economic globalization becomes more and more obvious, the professional knowledge of various positions is accelerated. The original knowledge and skills of many employees can no longer meet the needs of work. Short-term training and further study are provided by college education to enhance self-competitiveness [1]. Therefore, there is a huge market demand for skilled talents cultivated by college education [2]. From a theoretical point of view, although people are paying more and more attention to the mental health of college students, the attention to the special group of college students is far from enough. They both have the common psychological problems of contemporary college students [3–5]; at the same time, under the influence of the characteristics of college education, some more prominent psychological phenomena have emerged. Therefore, research on the mental health status of college students is particularly important [6], but most of the current research on the mental health status of college students is only based on theoretical analysis and rarely on the basis of data obtained through surveys [7].

However, the mental health prospects of college graduates are not optimistic [8]. While constructing and improving the quality of teaching, we should also pay attention to the cultivation and development of the comprehensive quality of college students, especially the healthy development of their psychological quality [9–11]. Therefore, it is necessary to pay attention to and study the physical and mental health development of college students. From a practical point of view, the university stage is an important turning point in the life of college students [12]. Since many of the problems that trigger test anxiety are imaginary, desensitization techniques can use the test taker's imagination to resist these stimuli. During this period, individuals will inevitably suffer from various pressures and discomforts [13]. Therefore, research on the mental health of college students can help school workers to grasp the psychological dynamics of students and help school workers to formulate more scientific and reasonable related policies to promote the mental health of college students [14].

This paper conducts a questionnaire survey, supplemented by case interviews, etc., to understand the current psychological status of college students, conduct statistical analysis of the survey results, and summarize the current problems and characteristics of college students' mental health. Through the analysis of the development characteristics of English test anxiety among middle school students of different genders, it can be seen from the data that boys and girls show basically the same development characteristics, which is also consistent with the development characteristics of the overall students. However, through the analysis of variance and further LSD multiple comparison results, it shows that there is no significant difference between the grades of college girls, because college girls are significantly higher than boys in terms of self-esteem, self-education ability, and independence. Cognition and evaluation are the main reasons for English test anxiety, and the percentage of students who choose this item is as high as 68.1%; as external factors, family education, school education, and social environment are also important reasons for students' English test anxiety, and the percentages are 39.5%, 33.4%, and 26.5%; other factors also have a certain influence on students' English test anxiety and cannot be ignored. This is a chronic neurotic anxiety disorder, which shows that the test taker's fear and worry about the test have formed a vicious conditioned reflex, and an inexplicable fear of the coming of the test has occurred, indicating that the test taker's mental health has been affected. This paper starts with the questionnaire survey, through the actual survey, using data to speak, to provide theoretical support and data support for the research on the mental health of college students. Finally, the corresponding intervention measures are put forward to improve the mental health of college students, in order to provide useful guidance and help in improving the mental health of college students.

## 2. Related Work

With the development of society, the state pays more and more attention to college education, and the society pays more attention to the mental health of college students [15]. Many educators have set up a research project on the mental health development of college students and conducted special surveys, using more survey tools such as Self-Esteem Scale (SES), Psychological Symptom Self-Assessment Scale (SCL-90), and Mental Health Survey Scale; through these classic mental health tests, they believe that the psychological development of most college students in the region is healthy, and the overall psychological state is good, but there are still some psychological problems, mainly focusing on learning anxiety, communication confusion, and obsessive-compulsive tendencies [16].

The results of Fancourt and Tymoszuk's [17] study show that the achievement in reality of people with low self-evaluation will be greatly affected by failure feedback, and they will underestimate their future achievements; however, subjects with high self-evaluation are less susceptible to failure feedback, and they will overestimate their future achievements. People with high self-evaluation attribute their success to their own abilities and attribute their failure to external environmental factors, while people with low self-evaluation do the opposite. They think that their success is due to chance and good luck. Nahmias et al. [18] examined the explanations given by subjects of different genders on the success or failure of the task: no matter what the task, male subjects tend to attribute their good achievements to internal factors such as ability and skills. The female subjects' explanations for the reasons depended more on the nature of the task, and when they succeeded in the task, they did not show an obvious tendency to be their own trait. Many studies have shown that rational emotional therapy and rational system reconstruction can effectively alleviate English test anxiety but have no significant effect on the improvement of academic performance. Maramba et al. [19] proposed cognitive-attention training, which is intended to allow individuals to focus on task-related stimuli, thereby reducing resource allocation for English test anxiety.

Nyashanu et al. [20] conducted a comparative study on the relationship between psychology and mental health among foreign college students of different ethnic groups, and the results showed that different ethnic groups and cultures, attributes of luck to events, have poorer mental health level. In cognitive therapy, rational emotion therapy and rational restructuring of the system are commonly used techniques. Research by Fritz et al. [21] showed that students who explained their learning success as stable factors such as their own ability and perseverance had lower anxiety levels than those who explained their success as low-stable factors such as luck. There is a big difference between boys and girls in the distribution of English test anxiety levels. Boys have a higher proportion of low English test anxiety levels (19.4%) than girls (15.0%), while girls have high English test anxiety levels. The proportion (17.2%) is larger than that of boys (14.1%). The proportion of male and female students in the medium anxiety level is not much different, which are 66.5% and 67.8%, respectively. Students with high stability factors had higher anxiety levels than those explained by low stability factors such as insufficient effort and bad luck [22, 23].

## 3. Methods

### 3.1. Mental Health Level Classification

The mental health level adopts the prepared teacher-student relationship grade for middle school students, and the questionnaire adopts the form of Likert five-point scale. It includes four dimensions of avoidance *p*(*s*, *t*), conflict *p*(*s*), intimacy *p*(*t*), and attachment *p*(*s*|*t*). The higher the score is, the stronger the relationship between students and teachers is. Avoidance consists of 4 items; conflict consists of 9 items; intimacy consists of 4 items; and attachment consists of 5 items, for a total of 22 items.

(1) $$\begin{array}{c} \left\{\begin{array}{c} \partial p\left(s,t\right)\left\{y\left[\left(p\left(s\right)\times p\left(t\right)\right)+p\left(s\left|t\right.\right)\right]\right\}=p\left(t\right)\\ \partial p\left(t,s\right)*p\left(x\right)=p\left(s\right) \end{array}\right.. \end{array}$$

The scores of each subscale of different mental health interventions were significantly different (*P* < 0.001), and the scores of SCL subscales of different mental health interventions were significantly different except for hostility (*P* < 0.001, *P* < 0.01, or *P* < 0.05). Further LSD (least significant difference) test showed that the scores of each subscale of students with a large amount of mental health intervention were higher than those of students with a small amount of mental health intervention (*P* < 0.001) and higher than those of students with a central mental health intervention (*P* < 0.001, *P* < 0.01, or *P* < 0.05); the scores of SCL subscales of the students with a large amount of mental health intervention max(*p*(*s*)) were lower than those of the students with a small amount of mental health intervention (*P* < 0.001 or *P* < 0.01) and lower than those of the students with a medium amount of mental health intervention, but the difference *p*(*s*) − *p*(*t*) was not significant (*P* > 0.05). The total score of the scale is obtained by adding up the scores of each item in the scale and then correlating the score of each item with the score of the total scale to obtain the degree of discrimination of the item.

(2) $$\begin{array}{c} \frac{\partial p\left(s,t\right)}{\partial p\left(s\right)}=\arg\max\frac{\left(p\left(s\right)-p\left(t\right)\right)}{\partial p\left(s\right)}-\frac{p\left(s\left|t\right.\right)*p\left(t\right)}{\partial p\left(t\right)}. \end{array}$$

Except for autonomy, the scores of each subscale of students with mental health intervention were higher than those of students with small mental health intervention (*P* < 0.001 or *P* < 0.01) and the scores of SCL subscales of students with medium mental health intervention except for paranoia factor *s*(*m*)*t*(*m*). In addition, the scores of other factors were lower than those of students with a small amount of mental health intervention (*P* < 0.01 or *P* < 0.05). It shows that the mental health level of students with a large amount of mental health intervention is the highest, followed by students with a medium mental health intervention, and the mental health level of students with a small amount of mental health intervention is the lowest.

(3) $$\begin{array}{c} \arg\max\left(p\left(s\left|t\right.\right)*p\left(t\right)\right)=\left\{\begin{array}{c} \left\{\sum 1-p\left(s+x\right)\right\}\\ \left\{\sum s\left(m\right)t\left(m\right)\right\} \end{array}\right.. \end{array}$$

Academic achievement *p*(*s* + *x*) is the effectiveness of the coursework learned, usually expressed numerically. In this study, the academic performance will be standardized according to the grade of the subject, and the standard *T* score will be obtained, where *T* = 50 + 10(*s* − *t*)/*s*. The survey results of anxiety levels of different test contents show that the percentages of very anxious and general anxiety are added together, and their scores are arranged from large to small as follows: listening 59.0%, completion dialogue 54.3%, cloze 54.0%, reading comprehension 48.8%, written expression 25.9%, and single choice 22.7%. Judging from the test content, college students are more anxious about listening, completing dialogues, and cloze during the English test.

### 3.2. Pre-Exam Emotional Intervention

Emotional intervention *p*(*s*)∗*p*(*t*) before the test analyzes the relationship between students' preference for English classes and teaching methods; teaching content, teachers' abilities, and teaching effects (X1), the score of teaching content (X2), the score of teaching effect (X3), and the score of teachers' teaching ability (X4) are independent variables, and multiple linear regression analysis is carried out. Using the ENTER method, the results show that the four independent variables are all entered into the equation, the multiple correlation coefficient of the equation is 0.616, the coefficient of determination is 0.380, and the significance test of the regression equation is *P* < 0.001. They believed that the questionnaire basically covered various manifestations of test anxiety of middle school students and could effectively measure the test anxiety of middle school students; the topic is more representative.

(4) $$\begin{array}{c} p\left(s\left|t\right.\right)/p\left(s\right)*p\left(t\right)=p\left\{\lambda_{1},\lambda_{2},\lambda_{3},\cdots ,\lambda_{m-1},\lambda_{m}\right\}-p\left(t\right)p\left(s\right)/p\left(s,t\right). \end{array}$$

This equation *x*(*m*) shows that teaching methods, teaching content, teachers' abilities, and teaching effects are closely related to students' preference for English classes. The higher the scores of teaching method *y*(*m*), teaching content, teacher ability, and teaching effect, the higher the students' preference for English class. It is suggested that if you want to improve students' interest in English classes, teachers should start by improving teaching methods, teaching content, teachers' abilities, and teaching effects.

(5) $$\begin{array}{c} \exp\overset{m-1}{\underset{m=0}{\sum }}p\left(s,t\right)<x\left(m\right)\lambda_{i}\left(t,s\right)<y\left(m\right)h_{i}\left(t,s\right)\leq p\left(s\right)p\left(t\right). \end{array}$$

Avoidance mainly refers to students' avoidance of teachers in attitudes and behaviors and reluctance to communicate. Conflict refers to the inconsistency and disharmony of behavior and emotion between students and teachers. Intimacy refers to the intimacy and harmony between students and the classroom. Attachment refers to students' admiration for teachers and their attention to their attitudes and behaviors.

There is an extremely significant negative correlation between English test anxiety and all subscales of middle school students' mental health (MHS).  Figure 1 shows that English test anxiety affects five aspects of middle school students' mental health (cognition, emotion, will, personality, and adaptation). The results show that English test anxiety and cognitive normality (A) are significant negative correlations between the content scales in the English test anxiety and the 21 content scales in the MHS. Except for well-being (B4), there were significant negative correlations between English test anxiety and other content scales (B). There is an extremely significant negative correlation. English test anxiety is only significantly negatively correlated with the two content scales of activity (D2) and extraversion (D3) in personality integrity (D), while there is a significant negative correlation with conscientiousness (D1), and the correlation between independence (D4) did not reach a significant level. There were extremely significant negative correlations between English test anxiety and well-adjusted (E) content scales. According to the general principles of psychometrics, a score above 0.4 indicates good discrimination, an item below 0.4 but above 0.3 is considered to have good discrimination, and a score below 0.3 is considered poor discrimination.

The results showed that all SCL-90 factor scores had a stable and low degree of negative correlation with students' preference for English classes (*P* < 0.001); all subscale scores had a stable and low degree of positive correlation with students' preference for English classes. Correlation relationship is *P* < 0.001, suggesting that the more students love English classes, the better their mental health. This result also supports the hypothesis that physical exercise promotes mental health from another aspect.

### 3.3. Analysis of Psychological Related Factors

The research on psychological related factors adopts the method of random sampling, randomly selects students of grades as the research objects, and selects 5 key classes and ordinary classes for investigation, taking the class as the unit, under the organization of the psychology teacher, using the self-study class time to use unified guidance. The students were tested by language and questionnaire, and the whole test took 45 min. 315 questionnaires were actually distributed; 295 questionnaires were recovered; the recovery rate was 93.7%; 293 valid questionnaires were obtained, and the effective rate was 93%. The evaluation of the teaching situation of English courses in colleges and universities for the English test shows that the students' scores on the teaching methods, teaching contents, teaching effects, and teachers' abilities of English courses are 7.34, 7.33, 7.05, and 80.70 (percentage system), respectively.

In order to ensure the representativeness of the sample, the method of stratified sampling was adopted in the test, and twelve classes of students (from the first grade to the third grade of senior high school) were selected from four middle schools in the city (including two key middle schools and two ordinary middle schools).

Figure 2 carries out variance analysis on the mental health (MHS) of middle school students with different English test anxiety levels. The results show that there are extremely significant differences in mental health scores (*P* < 0.01). With the increase of English test anxiety, students' mental health scores are, in turn, 251.97, 232.74, and 194.05. Such repeated training enables the candidate to gradually successfully adapt to each stimulus and is no longer sensitive to any stimulus that causes anxiety, until the strongest stimulus still fails to arouse the respondent's anxiety, and desensitization is successful.

A questionnaire survey on 128 students uses SCL-90 scale, English activity level scale, English exercise feeling scale, self-made physical education questionnaire, etc.; there are obvious gender differences in the mental health level of English test students, which is that the mental health level of boys is higher than that of girls; psychological problems of rural students are more than urban students; English majors have significantly higher levels of mental health than liberal arts and science students and are also better than liberal arts and science students in terms of fear factor, and science students are better than liberal arts students in terms of self-acceptance and identity; students in high grades were better than students in lower grades in the dimensions of autonomy, environmental adaptation and control, self-acceptance and identification, obsessive-compulsive symptoms, and psychosis. But this kind of tension will not affect the students' normal diet, sleep, and review before the exam, and it will stop naturally with the end of the exam. This kind of anxiety is generally useless for exams.

## 4. Results

### 4.1. Evaluation of Mental Health Effects

A total of 300 questionnaires were distributed, and 277 valid questionnaires were recovered, with a recovery rate of 92.3%. After excluding 20 invalid questionnaires, 257 valid questionnaires were obtained, with an effective rate of 85.7%. The scale includes ten items, which are scored from positive and negative directions. The score range is generally between 10 and 40. In this study, the Cronbach coefficient of the scale was 0.7952, indicating good validity. Further test (LSD method) showed that, except for the sense of goal and direction (*P* > 0.05), English majors were significantly different from liberal arts students in the above dimensions (*P* < 0.01); English majors were significantly different in the above dimensions. There is a significant difference with science students in dimensions (*P* < 0.05), indicating that in the above dimensions of mental health, English majors are better than liberal arts and science students; in the dimensions of self-acceptance and identity, science students are better than liberal arts students (*P* < 0.05).

The results of variance analysis in Table 1 on the academic performance of middle school students with different English test anxiety levels show that there are significant differences in the academic performance of students with different English test anxiety levels (*P* < 0.05).

Compared with the comprehensive sample of college students, the average of the nine factors of SCL-90 of college students is also higher than the indicators in the comprehensive sample of college students, *P* < 0.001. Compared with most colleges and universities in the country, the relatively pure university culture of English-speaking colleges and universities increases the closed limitations and development lag of students, resulting in extreme cognitive biases and obstacles to the development of self-consciousness among college students. The Cronbach's alpha coefficients of positive events and negative events analyzed by verbally explained content technology are 0.8 and 0.89, respectively. Taking the attribution analysis of negative event subscales as an example, the three dimensions of self, wholeness, and persistence were cloned. The coefficients are 0.93, 0.48, and 0.63, respectively.

### 4.2. Analysis of English Test Experiment Variables

The mental health test scale (MHT) for college students contains eight content scales and one validity scale (i.e., the polygraph scale). In this survey, the Cronbach coefficient of the validity scale (i.e., the polygraph scale) was 0.921, and the Cronbach coefficient of each subcontent scale was 0.689–0.784, indicating good construct validity. In terms of autonomy, successful experience and sense of control, empathy, and cooperation, *P* < 0.01; in the dimensions of goal and sense of direction, *P* < 0.05; the results show that, except for terrorist factors, there was no significant difference in the scores of literature, science, and physical education among the SCL-90 factors.

It can be seen that there is an extremely significant negative correlation between English test anxiety and academic performance and mental health (*r* = −0.219, *r* = −0.442), and there is a significant positive correlation between mental health and academic performance (*r* = −0.219, *r* = −0.442). This shows that on the whole, the higher the level of English test anxiety, the worse the students' academic performance and the worse their mental health; and the better the students' mental health, the higher the students' academic performance. The characteristics of the development of grades increase, and the causes of test anxiety are also discussed, in order to provide a basis for the development of school teaching and mental health work in middle schools.

The statistical results in Figure 3 show that college students' psychology and academic performance are 0. There is a significant correlation at the 0.5 level (two-sided), which also shows that psychology has an impact on students' academic achievement. Generally, students with higher academic achievement are more optimistic, while students with lower academic achievement tend to be more “pessimistic”. There are differences in the mental health status of college students of different grades, but the difference is not significant. Freshmen and juniors have higher psychological anxiety, especially juniors. Sophomores had the lowest levels of anxiety. The psychological anxiety factors of freshmen and juniors are different. Freshmen have just entered the school and are in the process of changing from the middle school learning mode to the university learning mode. In addition, the changes in the campus environment and interpersonal environment have brought them. Among them, there are 3 key middle schools and 3 ordinary middle schools, each with 6 classes and 3 classes in each grade, for a total of 18 classes. After the questionnaire was withdrawn, 32 invalid questionnaires were excluded, and 727 valid questionnaires were obtained. For the distribution characteristics of the subjects, see the article.

## 5. Discussion

### 5.1. Analysis of Mental Health Relationship

After inputting the mental health assessment data into the computer, SPSS for Windows 10.0 statistical software was used to analyze and process the data. The scale used in this study was revised based on Zimct's Perceived Social Support Scale. Considering that the test subjects were students, the “colleagues and leaders” in the original scale were replaced with “classmates and teachers”. The scale has 12 self-assessment items, of which “family support” is scored by 3, 4, 8, and 11 questions, “friends' support” is scored by 6, 7, 9, and 12 questions, and “others' support” is scored of questions 1, 2, 5, and 10. The cumulative score of all questions is the total score of social support. If the total score of social support is less than 50 points, it means that there is a problem with the student's social support; if the score of this item is less than 32 points, it shows that the student has serious defects in social resources and social support system.

There are four dimensions of positive high arousal, positive low arousal, negative high arousal, and negative low arousal. Positive high arousal has 8 items, including pride, joy, and hope; positive low arousal has 6 items, including calm and relaxation; negative high arousal has 8 items, including irritability, worry, hate, and shame; negative low arousal has 12 items, including boredom.

The test-retest reliability of Figure 4 is 0.79 (*P* < 0.01), and the test-retest reliability of each subscale of A, B, C, D, and E are 0.70, 0.77, 0.70, 0.72, and 0.72 (*P* < 0.01), respectively. The split-half reliability of the overall scale was 0.71 (*P* < 0.01), and the Cronbach alpha coefficient of consistency was 0.75 (*P* < 0.01). The scale has high criterion validity; the correlation coefficient with SCL-90 is 0.65 (*P* < 0.01); the correlation with the mental component of CMI is 0.72 (*P* < 0.01), and the correlation with 16PF psychological factors is 0.72 (*P* < 0.01). For the convenience of research, this study did not adopt these scales, but based on the abovementioned scales and interviews with teachers and students, firstly, according to the symptoms of test anxiety, it was divided into psychological symptoms and physical symptoms. The scale has good construct validity, indicating that the fitting degree of the structural model is good. The scale has a standardized norm for the mental health level of middle school students and divides the mental health status of middle school students into five grades from low to high: very poor, poor, medium, upper-middle, and excellent.

In terms of the scores of each factor of SCL and the average score of SCL, except for the somatization factor, the scores of other eight factors, and the average score of SCL, the scores of urban students are lower than those of rural students (*P* < 0.001), which indicates that rural students have more psychological problems for urban students. The reason may be that urban students adapt more quickly to university life and have stronger self-confidence. The overall mental health of girls is slightly lower than that of boys; especially in terms of “communication confusion tendency” and “depression tendency”, there are significant differences between boys and girls. Boys are slightly higher than girls in “impulsive tendency”, “horror tendency”, and “sexual tendency”, but the difference is not obvious. Some subjects were tested one week before the mid-term exam and one week before the final exam in the same semester, and the time interval was two and a half months. The test-retest reliability of the scale was 0.849 (*P* < 0.01). According to the requirements of psychometrics, the reliability coefficient above 0.70 is acceptable. It can be seen that this scale has good test-retest reliability.

### 5.2. The Degree of Emotional Control

The independent variable of the experiment is the emotional control of teacher-student relationship; the dependent variable is the academic emotion and student achievement, and the unrelated variables are mainly controlled by the balance method and the constant method. The experimental class and the control class are taught by the same teacher, and the teaching content, teaching hours, teaching progress, teaching venue, and teaching environment (such as area, light, noise, temperature, and humidity) are basically the same. The content of the intervention is based on positive psychology and communication analysis theory. Teachers' intervention methods are lectures and communication counseling; students' intervention methods are a combination of mental health group counseling and individual counseling. Only the experimental class was intervened, and the control class was taught according to the original teaching plan. The main tester of each class was a psychology graduate student. The instructions for administering the English test anxiety are the same as above, and the instructions for administering the MHS test can be found. The questionnaires were collected on the spot after the test was completed, and the test time was about 45 min.

The data showed that there was no difference in the four dimensions of academic emotion between the experimental class and the control class before the experiment. After the experiment, the scores of the students in the experimental class in positive academic emotions were higher than their pretest scores, and the scores in negative academic emotions were lower than their pretest scores. However, there was no significant change in the pretest and post-test scores of academic mood in the control class.

However, it does not reflect the specific relationship between the three, such as the impact of different test anxiety levels on the academic performance and mental health of middle school students, the impact of test anxiety on mental health, the relationship between different mental health levels and academic performance, and so on. Communication confusion tendency. College students yearn for friendship and expect to gain understanding and emotional support through interpersonal communication. However, they also lack interpersonal skills and skills to deal with interpersonal conflicts, and it is difficult to establish close relationships with others. It is this strong gap between high expectations and low results that makes college students prone to low self-esteem, self-isolation, and a strong sense of loneliness. Obsessive-compulsive tendencies. The main manifestations are compulsive thoughts and compulsive actions. Some students clearly know that a certain idea is wrong, but they cannot help thinking about it often, and they clearly know that a certain action has been completed, but they still cannot control to repeat the action repeatedly.

### 5.3. Example Application and Analysis

In this study, SPSS 11.5 software was used to process the data obtained from the survey, and the data was entered and aggregated for analysis. The main statistical analysis methods used were as follows: (1) *T* test: used to compare different family backgrounds, whether the only child and other factors have an impact on the psychological status of college students; (2) analysis of variance: used to analyze and compare the factors that affect the psychological status of college students (such as grades and family emotional status); (3) descriptive statistical analysis: mainly used to summarize the overall situation of the psychological state of college students; and (4) Spearman correlation analysis: used to study the correlation between individual social support status and mental health status. Then, according to the different learning periods of middle school students, it is divided into several dimensions: usually, before the test, during the test, and after the test, and compile the questions based on the performance of these two aspects.

The scores of several subscales of the scale and the total score were higher than those of girls (*P* < 0.001), in the comparison of each factor score of SCL-90 and the average score of SCL, except for the three factors of hostility, paranoia, and psychosis. In addition to no difference between men and women, there were differences between men and women in the other six factors and the average score of SCL (*P* < 0.001). In addition, women's menstrual cycles have a certain fluctuating effect on mental health. However, even if tension is widespread, the resulting symptoms are not necessarily recognized by the individual, so it is normal that there are no differences between men and women in hostility, paranoia, and psychosis.

The data in Figure 5 show that both attachment and intimacy in the teacher-student relationship are significantly positively correlated with positive high arousal and positive low arousal academic emotions and significantly negatively correlated with negative low arousal academic emotions. Both conflict and avoidance were positively correlated with negative high arousal and negative low arousal academic emotions and negatively correlated with positive high arousal and positive low arousal academic emotions. The mental health of only children is significantly better than that of non-only children. The only child is the focal point of the family, and they can receive more material and spiritual support than non-only children. Too high expectations can easily lead to tension before the test and frustration after the test, which can cause students to react to test anxiety; too low expectations will make students lack the necessary motivation and reduce their enthusiasm for learning.

Analysis of variance was conducted on the academic performance of students with different mental health levels, and the results showed that there was an extremely significant difference in academic performance (*F* = 5.084, *P* < 0.01). Although the average score of the students in the “excellent” grade is lower than that of the students in the “upper middle” grade, the difference between the two is not significant (*P* = 0.227), so the overall trend is that the higher the mental health grade, the higher the academic performance score. This is also consistent with the result. When encountering difficulties in life and study, strong family support will help them effectively relieve stress. Literature and history students have the highest anxiety and the worst mental health, followed by art students, and finally science and engineering students. Through postmortem examination, it is found that the psychological anxiety of students majoring in literature and history is significantly higher than that of students majoring in science and engineering and students majoring in art. Therefore, the mental health of college students is affected by the majors they study, but the difference is not significant.

## 6. Conclusion

The results of this study show that there is a significant positive correlation between mental health and academic performance of college students in general. Except for perceived awareness, mild excitement, well-being, extroversion, spiritual coherence, and interpersonal relationships, other factors of mental health are related to academic performance. There is a significant positive correlation between academic performance and various subscales of mental health; the results of the correlation between academic performance and various content scales show that there is a positive correlation between academic performance and 21 content scales of mental health, except for perceptual awareness. By analyzing the various factors in the mental health scale, it can be seen that, in addition to the abovementioned factors that are not significantly related to academic performance, the main intellectual factors such as understanding, judgment, and reasoning in the cognitive dimension of mental health have a direct impact on academic performance. This is especially beneficial for clients with social skill impairments, as they can learn to adopt more beneficial behaviors by getting feedback from children and group leaders about the effects of their interpersonal behaviors, while the factors included in the dimensions of emotion, personality, and social adaptation belong to the category of nonintellectual factors, which indirectly affect academic performance through the regulation of intellectual activities. In addition, it will also have a negative impact on the development of their own emotions, will, personality, and social adaptation.

## Figures and Tables

**Figure 1:** Emotional intervention model before the test.

**Figure 2:** Significant difference analysis of psychological related factors.

**Figure 3:** Statistical error distribution of English test experimental variables.

**Figure 4:** Test-retest reliability analysis of mental health relationship.

**Figure 5:** Correlation distribution of students' academic mood and test scores.

**Table 1:** Analysis of mental health effects.

Mental node	Coefficient *a*	Coefficient *b*	Coefficient *c*	Coefficient *d*	Coefficient *e*
10	0.49	0.27	0.03	0.00	0.28
20	0.97	0.59	0.13	0.01	0.40
30	0.63	0.80	0.84	0.04	0.86
40	0.66	0.46	0.70	0.04	0.59
50	0.03	0.62	1.00	0.05	0.27

## Data Availability

The data used to support the findings of this study are available from the corresponding author upon request.
